# Synergistic Effect of Polydatin and *Polygonatum sibiricum* Polysaccharides in Combating Atherosclerosis via Suppressing TLR4-Mediated NF-*κ*B Activation in ApoE-Deficient Mice

**DOI:** 10.1155/2022/3885153

**Published:** 2022-07-07

**Authors:** Genyi Ye, Yuhao Zhao, Junfeng Zhu, Zijian Zhang, Qiong Wang, Xu Jiang, Zhenxing Wang

**Affiliations:** ^1^Affiliated Hospital of Nanjing University of Chinese Medicine, Nanjing 21009, China; ^2^Pharmacology Laboratory, Jiangsu Province Hospital of Chinese Medicine, Nanjing 21009, China; ^3^Department of Science and Technology, Affiliated Hospital of Nanjing University of Chinese Medicine, Nanjing 21009, China; ^4^Department of Cardiology, Affiliated Hospital of Nanjing University of Chinese Medicine, Nanjing 21009, China

## Abstract

**Objective:**

Atherosclerosis is a chronic inflammatory disease, which is closely related to hyperlipidemia, inflammatory responses, and oxidative stress. As natural products, polydatin (PD) and *Polygonatum sibiricum* polysaccharides (PSP) have remarkable pharmacological effects in anti-inflammatory, antioxidant stress, and lipid regulation. In this study, we sought to investigate whether the combination of polydatin and *P. sibiricum* polysaccharides play an anti-atherosclerotic role in alleviating inflammatory responses by inhibiting the toll-like receptor4 (TLR4)/myeloid differentiation factor88(MyD88)/nuclear factor-kappa B(NF-*κ*B) signaling pathway.

**Methods:**

Thirty-two ApoE-/- mice were fed with a high-fat diet (HFD) starting at the age of 8 weeks. Mice were randomly divided into four groups; (1) model group, (2) PD (100 mg/kg) + PSP (50 mg/kg) group, (3) TAK-242 (3 mg/kg) (TLR4 inhibitor) group, (4) PD (100 mg/kg) + PSP (50 mg/kg) + TAK-242 (3 mg/kg) group. Eight age-matched wild-type C57BL/6J mice fed an ordinary diet were used as a control group. Blood lipid levels were measured with an automatic biochemical analyzer. The lipid accumulation and histopathological changes in the aorta and liver were observed by Oil Red O and hematoxylin and eosin (H&E) staining, respectively. ELISA was performed to measure the serum levels of vascular cell adhesion molecule-1 (VCAM-1) and intercellular adhesion molecule-1 (ICAM-1). Western blot analysis was performed to analyze the expression of key proteins in the TLR4/MyD88/NF-*κ*B signaling pathway.

**Results:**

Compared with the model group, the combination of PD and PSP significantly inhibit serum lipids (low-density lipoprotein cholesterol, total cholesterol, and triglyceride) and cell adhesion molecules (VCAM-1, ICAM-1). Oil Red O staining indicated that the combination of PD and PSP decrease lipid accumulation in the aorta and liver. Moreover, H&E staining suggested that the combination of PD and PSP alleviate aortic intimal hyperplasia, inflammatory cell infiltration, and hepatic steatosis. Finally, the combination of PD and PSP inhibit the expression of TLR4, MyD88, and the phosphorylation level of NF-*κ*B p65 protein in the aorta.

**Conclusions:**

Polydatin synergizes with *P. sibiricum* polysaccharides in preventing the development of atherosclerosis in ApoE–/– mice by inhibiting the TLR4/MyD88/NF-*κ*B signaling pathway.

## 1. Introduction

Atherosclerosis is the main pathological basis of cardiovascular and cerebrovascular diseases [1] that affect the quality of life that contribute to heavy economic burden. Lipid-lowering chemical agents play an important role in the treatment of atherosclerosis, especially statins that significantly reduced the level of low-density lipoprotein and atherosclerotic cardiovascular events. However, various toxic effects of these drugs have been confirmed, including stomach upset, liver dysfunction, myopathy, tickle, and rubefaction [2]. Natural product have good pharmacological properties and few side effects, they may serve as a novel therapeutic approach for the prevention and treatment of atherosclerosis and cardiovascular diseases.

Natural herbal products have long been applied in the treatment of myocardial ischemia-reperfusion injury, thrombosis, coronary artery disease, and atherosclerosis, and a growing evidence also supports their availabilities [3]. Polydatin (PD) is a primary active component from the roots of *Polygonum cuspidatum* Sieb. et Zucc, which has varied pharmacological properties, including antishock, regulation of blood lipids, lowering of cholesterol, anti-inflammation, and antiatherosclerotic properties [4]. Oxidative stress-mediated proliferation of vascular smooth muscle (VSMCs) was devoted to plaque formation and the progression of atherosclerosis. In a previous study, we found that PD inhibited the oxidative stress-induced proliferation of VSMCs by activating the endothelial nitric oxide synthetase (eNOS)/silent information regulator1 (SIRT1) pathway [5]. Moreover, polydatin could prevent atherosclerosis through enhancement of overall reverse cholesterol transport [6]. Autophagic restoration is a common regulatory mechanism that eliminates many atherosclerotic triggers. Recent studies have shown that Polydatin could enhance autophagy to alleviate atherosclerosis by inhibiting phosphoinositide 3-kinase (PI3K)/protein kinase B(Akt)/mammalian target of rapamycin (mTOR) [7]. However, there are still considerable uncertainties and challenges of the antiatherosclerosis mechanism of PD.

*Polygonatum sibiricum* polysaccharides (PSP) is one of the main bioactive components of *P. sibiricum*. PSP has many favorable therapeutic properties, such as immunity enhancement effect, antioxidant activity, anti-inflammatory effect, hypolipidemic, and antiatherosclerotic effects [8]. It has been reported that PSP can prevent lipopolysaccharide (LPS)-induced acute lung injury by way of inhibiting inflammatory responses via the TLR4/Myd88/NF-*κ*B signal pathway [9]. In addition, recent research has suggested that PSP may show a strong protective effect on gentamicin-induced acute kidney in rats by inhibiting the secretion of inflammatory factors via p38 mitogen-activated protein kinase (MAPK)/activating transcription factor 2 (ATF2) signal pathway [10]. As can be seen from the above, both PD and PSP have many common pharmacological properties, including anti-inflammation, regulation of blood lipids, antioxidant stress, and antiatherosclerosis effects. However, the antiatherosclerosis mechanism of the combination of PD and PSP is worthy of further exploration and research.

It has been reported that lipid metabolism disorders and inflammatory reactions play a crucial role in the pathological process of atherosclerosis [1]. It is also considered to be a chronic inflammatory disease affected by many factors, and inflammatory responses are involved in the whole process of atherosclerosis development [11].

TLR4/MyD88/NF-*κ*B signal pathway is one of the major emerging immunomodulatory and anti-inflammatory pathways [12]. TLR4, a typical pattern recognition receptor in innate immune responses that activates the transcription factor NF-*κ*B and leads to the production of proinflammatory cytokines. TLR4 signaling pathway has a vital role in lipid accumulation and inflammatory activation in atherosclerosis and is associated with atherosclerotic plaque vulnerability and progression [13]. The role of MyD88 and its association with TLRs in the development of atherosclerosis have been studied in ApoE–/–mice. Moreover, MyD88 deficiency has been shown to alleviate atherosclerotic lesions and the secretion of inflammatory cytokines [14]. A novel MyD88 inhibitor (LM9) can significantly reduce oxidative stress and vascular inflammation in mice, thus its inhibition can be considered as an effective target for the treatment of atherosclerosis [15]. The NF-*κ*B family of transcription factors plays an important role in innate immunity and inflammation [16]. Triggering the activation of the TLR4/NF-*κ*B signaling pathway leads to downstream proinflammatory responses that promote plaque instability and growth [17]. The high expression of vascular cell adhesion molecule-1 (VCAM-1) and intercellular adhesion molecule-1 (ICAM-1) promotes macrophage proliferation and results in a mass of macrophages accumulating in the plaque, increasing plaque instability [18]. It was reported that ICAM-1 is involved in the expression and formation of atherosclerotic plaques [19]. In patients at high risk of developing acute coronary syndrome, circulating VCAM-1 level may be associated with the extent of coronary lesions. Moreover, this result reveals that VCAM-1 may also be associated with the severity of atherosclerosis and the prediction of cardiovascular disease [20]. TLR4/MyD88/NF-*κ*B signaling pathway has been proved to be involved in a variety of pathological processes including inflammation, immune response, and cholesterol metabolism. Therefore, inhibition of this signaling pathway may become a new effective therapeutic target for atherosclerosis. TAK-242 effectively inhibited TLR4/MyD88/NF-*κ*B signaling pathway, reduced NOD-like receptor protein3 (NLRP3) inflammasome activation, and decreased the expression of tumor necrosis factor-*α* (TNF-*α*), interleukin-1*β* (IL-1*β*), interleukin-18 (IL-18), and other inflammatory cytokines [21].

In the present study, to clarify whether the combination of PD and PSP would have great effects on atherosclerosis, transgenic ApoE–/– mice model of atherosclerosis induced by HFD were used. We demonstrated that the combination of PD and PSP significantly inhibited serum lipids and cell adhesion molecules increase. Furthermore, we also found that the antiatherosclerotic effects of the combination of PD and PSP acted through inhibiting inflammatory responses via the TLR4/MyD88/NF-*κ*B signal pathway.

## 2. Materials and Methods

### 2.1. Experimental Animals

A total of 32 specific pathogen-free (SPF), 8-week-old male ApoE–/– mice (license no. SCXK (Jing) 2019-0010) and 8 age-matched wild-type C57BL/6J mice (license no. SCXK (Jing) 2019-0010) were purchased from SPF (Beijing) Biotechnology Co., Ltd. The mice were kept in the Animal Experiment Center of Nanjing University of Chinese Medicine. The room temperature was kept constant at 24 ± 1°C, the relative humidity was 40%–60%, the room was well ventilated, and the light was 10–12 hours a day. All mice had free access to food and water. The 8 weeks after the treatment period, all mice were fasted overnight. They underwent cervical dislocation after pentobarbital anesthesia to collect samples. All the experimental procedures were approved by the Experimental Animal Ethics Committee of the Affiliated Hospital of Nanjing University of Chinese Medicine (approval no. 2021DW-26-02). This study was conducted in accordance with the National Institutes of Health guidelines for animal care and use (published by the National Institutes of Health No. 85-23 Rev.1985).

### 2.2. Medicine and Major Reagents

TAK-242 (CAS Number: 243984-11-4; molecular formula, C_15_H_17_ClFN0_4_S; molecular weight, 361.82) was supplied by MedChemExpress Company (Princeton, NJ, USA). Polydatin (CAS Number: 65914-17-2; purity, 95%, molecular formula, C_20_H_22_O_8_; molecular weight 390.38) and Oil Red O (cat.no. 00625) obtained from Sigma-Aldrich (St. Louis, MO, USA). *P. sibiricum* polysaccharides (cat.no.A16GS145378, purity 70%) was obtained from Shanghai Yuanye Biotechnology Co., Ltd. The mouse ICAM-1 (cat.no. JYM0003Mo) and VCAM-1 (cat.no. JYM0251Mo) ELISA kits were purchased from Wuhan ColorfulGene Biological Technology Co., Ltd. Hematoxylin-eosin Dye kit (cat.no. KGAA224), Ecl chemiluminescence kit (cat.no. KPG1121), Rabbit Anti-GAPDH (cat.no. KGAA002), and HRP-linked anti-rabbit IgG (cat.no. KGAA35) were obtained from Jiangsu KeyGEN Biotechnology Co., Ltd. Rabbit Anti-TLR4 (cat.no. 19811-1-AP) was obtained from Proteintech (Rosemont, IL, USA). Rabbit Anti-MyD88 (cat.no. ab219413), Rabbit Anti-p65 (cat.no. ab32536), and Rabbit Anti-p-p65 (cat.no. ab76302) were supplied by Abcam (Cambridge, UK). Nitrocellulose (NC) membrane (cat.no.6648) was obtained from Pall (New York, USA).

### 2.3. Modeling and Grouping

After being fed with an ordinary diet for 1 week, 32 male, ApoE-/- mice were randomly divided into four groups by a random number table: (i) ApoE-/-mice + HFD (Model group); (ii) ApoE-/- mice + HFD + PD + PSP (PD + PSP group); (iii) ApoE-/- mice + HFD + PD + PSP + TAK-242 (PD + PSP + TAK-242 group); (iv) ApoE-/- mice + HFD + TAK-242 (TAK-242 group). Eight age-matched wild-type C57BL/6J mice fed an ordinary diet were regarded as a control group (WT group). The model group and wild-type group were intragastric with an equal amount of normal saline daily. HFD feeding to establish the atherosclerosis model and drug regimens started at the same time and lasted for 8 weeks. The HFD consisted of a normal mouse diet with an addition of 20% fat and 1.25% cholesterol. The behavior and health of the mice were monitored weekly. PD + PSP group was treated by daily oral gavage of a PD solution (100 mg/kg) [6] and a PSP solution (50 mg/kg) [9], and the TAK-242 group was treated by peritoneal injection of a water solution containing TAK-242 (3 mg/kg) [22] every other day.

### 2.4. Measurement of Serum Level of Blood Lipid

Mice were anesthetized by peritoneal injection of 0.05 ml, 2% pentobarbital sodium (50 mg/kg). The blood samples were collected before the mice were sacrificed by treating with cervical dislocation, and serum was prepared by centrifugation at 3000 rpm for 15 min. The automatic biochemistry analyzer (P800, Roche, USA) was used to detect the concentrations of total cholesterol (TC), triglyceride (TG), low-density lipoprotein cholesterol (LDL-C), and high-density lipoprotein cholesterol (HDL-C).

### 2.5. Histopathological Examination of Mouse Aortas and Livers

After perfusion fixation, aortas were opened longitudinally from brachiocephalic artery to iliac artery bifurcation. Aortas were fixed to a vessel and the peripheral fat and adventitial tissue were removed. The aortas were stained with Oil Red O solution. The images were captured with Bioluminescence microscope (BX41, Olympus, Japan). Moreover, the part of aorta ranging from the arch to the abdominal aorta and the liver were collected and fixed in 10% formaldehyde for the paraffin-embedded or frozen sectioning (−20°C). These tissue sections were used for hematoxylin and eosin (H&E) staining and Oil Red O staining. The histopathological examination of the mouse aortas and livers was observed under a Bioluminescence microscope.

### 2.6. Determination of Mouse Serum Levels of ICAM-1 and VCAM-1 Using ELISA

The mouse serum was prepared at first, and ELISA was performed according to the instructions. The serum levels of ICAM-1 and VCAM-1 were determined at OD_450_ nm and corresponded to the standard curves.

### 2.7. Western Blot Analysis of Protein Expression Levels of the TLR4/MyD88/NF-*κ*B Signal Pathway in Mouse Aorta

Total protein (30 *μ*g) per sample was loaded on 10% SDS-PAGE and transferred on to a nitrocellulose (NC) membrane. The membrane was blocked for 1 h with 5% skimmed milk in Tris-Buffered Saline Tween-20 and then incubated with 1 : 1000 primary antibody (TLR4, MyD88, NF-*κ*B p65, p-NF-*κ*B p65) at 4°C overnight, followed by secondary HRP-conjugated antibodies (1 : 2000). Protein expression was probed using Ecl chemiluminescence kit. Equal protein loading was normalized to GAPDH.

### 2.8. Statistics Analysis

The data were analyzed using SPSS 23.0 software (SPSS Inc., Released 2014. SPPS Statistics for Windows, Version23.0Armonk, NY, USA). The numerical data presented as the means ± standard deviation (‾*x* ± SD). Comparisons among multiple randomized groups were performed using one-way ANOVA, followed by LSD comparison between two groups. Differences were considered significant (*P* < 0.05) and very significant (*P* < 0.01). The data were plotted using GraphPad Prism 5 software (La Jolla, CA).

## 3. Results

### 3.1. Effect of the Combination of PD and PSP on Serum Lipid Parameters

Hyperlipidemia is a major risk factor for atherosclerosis and will accelerate the development of atherosclerosis, so the regulation of blood lipids has become an important strategy for the prevention of atherosclerosis. As shown in Figure 1, after 8 weeks of feeding on the HFD, ApoE–/– mice had significantly higher serum TC, TG, and LDL-C levels and lower serum HDL-C level compared with the WT group (*P* < 0.01). Compared to the model group, treatment with PD and PSP or TAK-242 significantly decreased the levels of TG, TC, and LDL-C and increased the level of HDL-C (*P* < 0.01). Moreover, the levels of TC and LDL-C were more significantly decreased in the PD + PSP + TAK-242 group. The results showed that PD and PSP maintained the lipid metabolism balance of ApoE–/– mice induced by HFD.

### 3.2. Effect of the Combination of PD and PSP on Atherosclerotic Lesion Formation

To solve the key problem of whether the combination of PD and PSP can protect blood vessel function and alleviate the formation of the atherosclerotic lesion. Oil Red O and H&E staining were used for the pathological analysis. It was intuitively plausible that the aorta of the WT group was smooth and clean, that of the model group had more obviously lipid droplets, and the other groups using PD, PSP, and/or TAK-242 had fewer lipid droplets than the model group to some extent (Figures 2(a) and 2(b)). Further observation of H&E staining of aortas was shown in Figure 2(c). The WT group had intact arterial vascular structure and elastic fiber structure without inflammatory cell infiltration. In the model group, vascular intima hyperplasia was obvious, inflammatory cells were infiltrated, and elastic fiber structure was disorder. Compared to the model group, the other groups all seemed to improve the regional damage of atherosclerotic lesions in the aorta. From the above, it is indicated that the combination of PD and PSP can reduce the degree of atherosclerotic lesions.

### 3.3. Effect of the Combination of PD and PSP on HFD-Induced Hepatic Steatosis

At the end of 8 weeks, HFD-fed ApoE–/– mice exhibited pale yellow livers indicating lipid accumulation in the liver (Figure 3(a)). Oil Red O staining revealed that lipid droplets were distributed sparsely throughout the hepatic tissue in the WT group. Compared with the WT group, there was the obvious accumulation of lipid droplets with varied shapes and sizes in the liver cell of the model group, and they were widely distributed. The number of hepatocytes with lipid droplets in the other three groups decreased (Figure 3(b)). The above results were further confirmed by H&E staining. H&E staining results of the liver show that mice in the WT group had a normal hepatic ultrastructure and without hepatocyte steatosis and inflammatory cell infiltration. By contrast, the mice in the model group had disorganized hepatic lobule structure. Hepatic cells were steatosis, inflammatory cells were scattered around the blood vessels hepatic lobule, and liver parenchyma. In PD + PSP, PD + PSP + TAK-242, and TAK-242 groups, liver damage was more improved than the model (Figure 3(c)). The combination of PD and PSP significantly improved hepatocyte steatosis, inflammatory cell infiltration, and the accumulation of lipid droplets in the liver cell.

### 3.4. Effect of the Combination of PD and PSP on the Levels of Cell Adhesion Molecules

Inflammatory responses are involved in the whole process of atherosclerosis development. Adhesion molecules have a critical role in the development of atherosclerotic plaques. Compared with the WT group, the levels of ICAM-1 and VCAM-1 in ApoE–/– mice were significantly increased (*P* < 0.01). Compared to the model group, treatment with PD and PSP or TAK-242 significantly decreased the levels of ICAM-1 and VCAM-1 (*P* < 0.01). The level of VCAM-1 in the PD + PSP + TAK-242 group was significantly lower than the levels of the PD + PSP and TAK-242 groups (*P* < 0.05) (Figure 4). In short, the combination of PD and PSP effectively inhibited the secretion of inflammatory cell adhesion molecules, thus alleviating inflammatory responses.

### 3.5. Effect of the Combination of PD and PSP on the Expression of the TLR4/MyD88/NF-*κ*B Signal Pathway in Aorta

To elucidate the potential molecular mechanism of the anti-inflammatory effect of the combination of PD and PSP, we evaluated the expression of key proteins in the TLR4/MyD88/NF-*κ*B signaling pathway in aorta fractions by western blotting. The protein expression levels of TLR4 and MyD88 in the model group were higher than those of the WT group (*P* < 0.01). In addition, the phosphorylation level of NF-*κ*B p65 protein was also increased (*P* < 0.01). Compared with the model group, treatment with PD, PSP, and/or TAK-242 significantly inhibited TLR4, MyD88, and the phosphorylation level of NF-*κ*B p65 proteins. All these protein levels in the PD + PSP + TAK-242 group were significantly lower than the levels of the PD + PSP and TAK-242 groups (*P* < 0.05) (Figure 5). The results suggested that the combination of PD and PSP could inhibit the activation of the TLR4/MyD88/NF-*κ*B signaling pathway.

## 4. Discussion

The pathogenesis of atherosclerosis is characterized by rapidly increasing inflammatory responses and lipids accumulation [23]. Apolipoprotein (Apo) E is a protein in plasma and plays a critical role in lipids metabolism. It had been demonstrated that ApoE deficiency could lead to the accumulation of cholesterol-rich remnants in plasma and then induce atherosclerosis [24]. ApoE–/– mice has been confirmed as an animal model to develop obvious hypercholesterolemia, with elevated LDL level and decreased HDL level [25]. Moreover, ApoE–/– mice is widely used in the basic research for atherosclerosis because of their ability to display pathological features of human atherosclerosis. In ApoE–/– mice, the development of atherosclerosis is spontaneous, even when fed a normal chow-diet [26]. There is an entire spectrum of atherosclerotic lesions in ApoE–/– mice [27]. From 6 weeks of age, monocytes adhered to endothelial cells, and foam cell lesions could be detected after 8 weeks. After 15–20 weeks, intermediate lesions will appear, which mainly include smooth muscle cells and fibrous plaque composed of smooth muscle cells, extracellular matrix, and necrotic core covering fibrous cap [28]. In more advanced lesions, calcified lesions of fibrous fat nodules will appear, and the plaque will become more calcified over time [29]. The time course of lesion formation was significantly accelerated when fed a western diet [27]. In this study, atherosclerosis model was established by feeding mice HFD. We observed that the combination of PD and PSP markedly improved the levels of blood lipid and alleviated the atherosclerotic lesions of aorta and liver steatosis in mice. In addition, the combination of PD and PSP significantly inhibited the secretion of inflammatory cell adhesion molecules and the expression of key proteins of the TLR4/MyD88/NF-*κ*B signaling pathway. Our results strongly supported that the combination of PD and PSP played an antiatherosclerotic role by inhibiting inflammatory responses through TLR4/MyD88/NF-*κ*B signaling pathway (Figure 6).

As is well known, the high level of TC or LDL-C has been regarded as the primary cause of atherosclerosis and cardiovascular disease [30]. The increasing evidence has demonstrated that the risk of cardiovascular disease events and mortality can be reduced if the circulating concentrations of LDL-C were further decreased [31]. Therefore, homeostasis regulation by targeting the level of these lipids is considered to be the most promising strategy for the treatment of atherosclerotic vascular disease [32]. Studies have shown that the hypolipidemic activity of PSP is due to the regulation of TC, LDL-C, and lipoprotein (Lp(A) in an atherosclerosis model and can also reduce the intima foam cells number and inhibit endothelial cells proliferation to play an antiatherosclerotic role [33]. Previous studies have confirmed that Pre-B-cell colony-enhancing factor (PBEF) affected inflammation and lipid deposition in atherosclerosis. PD could inhibit atherosclerosis through PBEF mediated reduction of cholesterol deposition in macrophages [13]. A recent study indicated that PSP could play lipid-lowering and anti-inflammatory roles by activating the adenosine monophosphate-activated protein kinase (AMPK) signaling pathway, thus improving HFD-induced mouse obesity [34]. In this study, our results reveal that the levels of TG, TC, and LDL-C were increased and the level of HDL-C was decreased markedly in the serum of HFD-induced ApoE–/– mice. However, after treatment with PD and PSP, this situation was reversed. The liver is an important organ regulating the homeostasis of lipid metabolism. In patients with atherosclerosis, the excessive increase of lipid levels, which exceeds the metabolic capacity of the liver, will damage the structure and function of the liver, resulting in hepatic steatosis [35]. Growing evidence has shown that hepatic steatosis is not only an indicator of atherosclerosis but also an early regulator to promote the development of atherosclerosis [36, 37]. Both atherosclerosis and hepatic steatosis, which is a lipid storage disease, involve disturbances in lipid metabolism and ongoing inflammatory responses. The further development of hepatic steatosis can lead to the aggravation of liver function damage. Hepatic dysfunction can accelerate the progress of atherosclerosis through the deterioration of dyslipidemia, systemic inflammatory response, and redox imbalance [38]. Oil Red O staining results also indicated that the combination of PD and PSP decreased lipid accumulation in the aorta and liver. Our results were well consistent with the previous study [15]. Therefore, the combination of PD and PSP could effectively regulate blood lipid levels to prevent atherosclerosis.

It is well established that atherosclerosis itself is an inflammatory responses process and plays a decisive role in the formation of atherosclerotic cardiovascular disease (ASCVD) [39]. It has been demonstrated that endothelial dysfunction can be caused by inflammation. Endothelial dysfunction is identified as an early indicator of atherosclerosis and is characterized by the high expression of VCAM-1 and ICAM-1 [40]. Previous studies have confirmed that ICAM-1 plays a vital role in the pathogenesis of atherosclerosis and the influences of many risk factors may be also mediated through their effects on ICAM-1 [41]. It was verified that PSP could increase liver antioxidant enzyme activities. Recent reports have suggested that PD can inhibit the expression of ICAM-1 in endothelial cells, thereby preventing the excessive adhesion of monocytes and endothelial cells [42]. In addition, the combination of palmitoylethanolamide (PEA) and PD alleviated inflammatory responses and oxidative stress in vessel damage and remarkably reduced the expression levels of ICAM-1 and VCAM-1 [43]. Our results also show the combination of PD and PSP significantly inhibited the secretion of ICAM-1 and VCAM-1 in the serum of ApoE–/– mice induced by HFD, thus protecting blood vessels from inflammation. The results were further supported by H&E staining results of the aorta and liver.

TLR4 has a critical role in adaptive and innate immune responses. One of the most important molecular pathways is through the major adaptor protein, MyD88. The ligation of TLR4 ligands results in the recruitment of MyD88 and thus leads to the activation of NF-*κ*B and mitogen-activated protein kinases (MAPK), which prompt the expression of proinflammatory genes [44]. Considerable evidence has proved that the activation of TLR4 may result in increasing the production of local or circulating proinflammatory cytokines [45]. Previous studies have shown that TLR4 plays a vital role in the pathogenesis of intimal hyperplasia, atherosclerosis, and hypertension [46]. Therefore, inhibition of TLR4 reduce inflammation and delay the progression of atherosclerosis. It was reported that TAK-242 alleviated crush injury-induced acute kidney injury via inhibiting the TLR4/NF-*κ*B signaling pathways in rats [47]. NF-*κ*B transcription factors are the major regulators of inflammation and cell death in the pathogenesis of atherosclerosis. It can regulate the expression of some functional genes involved in the development of atherosclerosis [48]. In addition, NF-*κ*B has since emerged as the major regulator of immune homeostasis and inflammation [49]. Previously studies reported that PSP can exert an immunoenhancement effect against lung cancer through inhibiting the TLR4-MAPK/NF-*κ*B signaling pathways [50]. PD has been shown to exert potential protective effects on lipoteichoic acid (LTA)-induced injury and it may occur via the attenuation of reactive oxygen species and the TLR2- NF-*κ*B signaling pathways [51]. In this study, we further explore the expression of the key proteins in the TLR4/MyD88/NF-*κ*B signaling pathway. All the expression of key proteins levels in the model group were significantly increased compared with the WT group, PD and PSP treatment markedly reversed this situation. Most of the previous studies focused on the expression of some genes but ignored the inflammatory signal pathway and its downstream- and upstream-related factors. Collectively, our present study demonstrated that the combination of PD and PSP inhibited inflammatory responses and played an antiatherosclerotic role by downregulating the expression of key proteins in the TLR4/MyD88/NF-*κ*B signaling pathway. It would open a new field for the treatment of atherosclerosis and inflammatory diseases in the future.

## 5. Limitations

We also had limitations in the study. First, only TLR4 antagonist TAK-242 was used in our study, theoretically speaking, the results would be more convincing if TLR4 agonist was used in another group. Second, there might be other molecular mechanisms involved in the pathogenesis of atherosclerosis, which might interfere with the real experimental results.

## 6. Conclusion

Taken together, our study provides strong evidence that the combination of PD and PSP can improve lipid levels and inhibit inflammatory responses as well as playing an antiatherosclerotic role in ApoE–/– mice induced by HFD. The possible potential mechanism is the association to anti-inflammatory effects inhibiting the TLR4/MyD88/NF-*κ*B signaling pathway. The combination of PD and PSP may afford the basis for a novel therapeutic approach for the inhibition of inflammation, which is devoted to atherosclerosis development and progression.

## Figures and Tables

**Figure 1:** Effect of the combination of PD and PSP on lipid level in serum of HFD-induced atherosclerosis ApoE–/– mice: (a) statistical chart of TC; (b) statistical chart of HDL-C; (c) statistical chart of TG; (d) statistical chart of LDL-C. Data are presented as the mean ± standard deviation (n = 4). ^a^*p* < 0.01, compared to the WT group; ^b^*p* < 0.01, compared to the model group; ^c^*p* < 0.01, and ^d^*p* < 0.05, compared to the TAK-242 group; ^e^*p* < 0.01 and ^f^*p* < 0.05, compared to the PD + PSP group. TC: total cholesterol; TG: triglyceride; LDL-C: low-density lipoprotein cholesterol; HDL-C: high-density lipoprotein cholesterol.

**Figure 2:** Effect of the combination of PD and PSP on atherosclerotic lesion in HFD-induced atherosclerosis ApoE–/– mice: (a) images of Oil Red O staining of the whole aorta; (b) images of Oil Red O staining of the aorta sinus of the lesion (×200); (c) H&E staining of aortic tissue (×400). WT: wild-type C57BL/6 mice fed an ordinary diet; model: ApoE–/– mice fed with high-fat diet; PD + PSP : ApoE–/– mice fed with high-fat diet, and treatment with PD and PSP; PD + PSP + TAK-242: ApoE–/– mice fed with high-fat diet, and treatment with PD, PSP, and TAK-242; TAK-242: ApoE–/– mice fed with high-fat diet, and treatment with TAK-242. PD : Polydatin; PSP : *P. sibiricum* polysaccharides.

**Figure 3:** Effect of the combination of PD and PSP on HFD-induced hepatic steatosis in ApoE–/– mice: (a) liver photos; (b) images of liver sections stained with Oil Red O (×200); (c) images of liver sections stained with H&E (×400).

**Figure 4:** Effect of the combination of PD and PSP on the levels of cell adhesion molecules in serum of HFD-induced atherosclerosis ApoE–/– mice: (a) statistical chart of ICAM-1; (b) statistical chart of VCAM-1. Data are presented as the mean ± standard deviation (*n* = 3). ^a^*p* < 0.01, compared to the WT group; ^b^*p* < 0.01, compared to the model group; ^c^*p* < 0.01 and ^d^*p* < 0.05, compared to the TAK-242 group; ^e^*p* < 0.01 and ^f^*p* < 0.05, compared to the PD + PSP group. ICAM-1: intercellular adhesion molecule-1; VCAM-1: vascular cell adhesion molecule-1.

**Figure 5:** Effect of the combination of PD and PSP on protein expression of TLR4, MyD88, p-p65, and p65 in aorta of HFD-induced atherosclerosis ApoE–/– mice: (a) TLR4, MyD88, p-p65, p65, and GAPDH expression exposed in WT group, model group, PD + PSP group, PD + PSP + TAK-242 group, TAK-242 group; (b) statistical chart of TLR4; (c) statistical chart of p-p65/p65; (d) statistical chart of MyD88. Data are presented as the mean ± standard deviation (*n* = 3). ^a^*p* < 0.01, compared to the WT group; ^b^*p* < 0.01, compared to the model group; ^c^*p* < 0.01 and ^d^*p* < 0.01, compared to the TAK-242 group; ^e^*p* < 0.01 and ^f^*p* < 0.05, compared to the PD + PSP group.

**Figure 6:** A proposed mechanism of synergistic effect of polydatin and *P. sibiricum* polysaccharides in combating atherosclerosis in ApoE–/– mice.

## Data Availability

The original contributions presented in the study are included within the article and further details can be obtained from the corresponding author upon request.
